# The effect of the efflux pump inhibitor Carbonyl Cyanide m-Chlorophenylhydrazone (CCCP) on the susceptibility to imipenem and cefepime in clinical strains of *Acinetobacter baumannii*

**DOI:** 10.1371/journal.pone.0259915

**Published:** 2021-12-17

**Authors:** Alejandra Sanchez-Carbonel, Belén Mondragón, Nicolás López-Chegne, Isaac Peña-Tuesta, Gladys Huayan-Dávila, Dora Blitchtein, Hugo Carrillo-Ng, Wilmer Silva-Caso, Miguel Angel Aguilar-Luis, Juana del Valle-Mendoza

**Affiliations:** 1 School of Medicine, Research and Innovation Center of the Faculty of Health Sciences, Universidad Peruana de Ciencias Aplicadas, Lima, Peru; 2 Servicio de Patología Clínica, Hospital Regional de Cajamarca, Cajamarca, Peru; 3 Laboratorio de Biologia Molecular, Instituto de Investigación Nutricional, Lima, Peru; Nitte University, INDIA

## Abstract

**Introduction:**

In the last years the rapid expansion of multidrug-resistant *A*. *baumannii* strains have become a major health problem. Efflux pumps are a group of transport proteins that contribute to the development of antibiotic resistance. The aim of this study was to evaluate the effect of the efflux pump inhibitor carbonyl cyanide 3-chlorophenylhydrazone (CCCP) on the antimicrobial action of imipenem and cefepime on clinical strains of *A*. *baumannii*.

**Materials and methods:**

A total of 49 non-duplicate clinical samples were collected during January through December of 2018 from patients hospitalized in the *Hospital Regional Docente de Cajamarca*. Of the 49 samples obtained, the confirmatory identification of *A*. *baumannii* was performed on 47 samples by molecular methods. The amplification of the bla*OXA-51-like gene* was carried out by polymerase chain reaction (PCR). The determination of the minimum inhibitory concentration (MIC) was calculated using the microdilution method in culture broth. The susceptibility to both antibiotics (cefepime and imipenem) was evaluated in the presence and absence of the inhibitor carbonyl cyanide 3-chlorophenylhydrazone (CCCP).

**Results:**

A total of 47 strains of *A*. *baumannii* were isolated: 97.87% (46/47) were resistant to Imipenem, 2.13% (1/47) of them were classified as intermediate and none of these strains were susceptible. On the other hand, 51.06% (24/47) of isolates were resistant to cefepime; 19.15% (9/47) intermediate and 29.79% (14/47) susceptible. We considered a significant difference in antibiotic susceptibility if the MIC changed at least 4 dilutions, after the addition of the inhibitor. In the case of CCCP in addition to imipenem, 2.1% (1/47) had a significant change of 4 or more reductions in MIC, 59.6% (28/47) achieved a change equal or less than 3 dilutions and 17.0% (8/47) did not have any change. In the case of CCCP with cefepime the percentage of strains with the significant change of MIC was 8.5% (4/47). On the other hand, 53.2% (24/47) presented a reduction equal or less than 3 dilutions and 12.8% (6/47) did not show changes.

**Conclusion:**

In conclusion, our results demonstrate that the use of CCCP may improve the antibiotic effect of imipenem and cefepime on clinical strains of *A*. *baumannii*. The relevance of this study is that it provides evidence that this efflux pump inhibitor may be an alternative treatment against multidrug-resistant *A*. *baumannii*.

## Introduction

*Acinetobacter baumannii* is a gram-negative opportunistic pathogen that causes 2–10% of all hospital-acquired gram-negative infections [1]. This pathogen is implicated in a great variety of nosocomial infections, including respiratory tract, bloodstream and urinary tract infections, being ventilator-associated pneumonia and bloodstream infections the ones with the highest mortality rates [2]. Infections are more common in immunocompromised patients such as the elderly, patients in the intensive care unit (ICU) or undergoing undergoing major invasive procedures, moreover it has been associated with extended periods of hospital stay [1, 3]. The epidemiological importance of this pathogens is due to the devastating outcomes associated with the infection such as mortality rates as high as 50%, its ability to survive for prolonged periods in surfaces around the patients and the emergence of multidrug-resistant strains [3–5].

In the last years the rapid expansion of multidrug-resistant *A*. *baumannii* strains has raised the medical and scientific community attention. In fact, the World Health Organization (WHO) released a list of microorganisms for which the development of new antibiotics is urgently needed, including *A*. *baumannii* among the group of highest priority [5, 6]. Also, the *Infectious Diseases Society of America (IDSA)* has considered this bacteria among the most important nosocomial infections worldwide, as it remains one of the most difficult to treat pathogens [7]. Previous studies from Latin America report that the prevalence of carbapenem-resistant *Acinetobacter spp*. is one of the most rapidly increasing in the world. For example, between the years 2000 to 2009 there were no cases of carbapenem-resistant strains in Peru [8]; however, in year 2013 the prevalence was 78% [9].

The high rates of antibiotic resistance have been attributed to three main mechanisms developed by this pathogen: enzymes that inactivate antibiotics, alteration of the target sites of antibiotics and reduction of antibiotics entry to the target site [10]. Efflux pumps are a group of transport proteins that contribute to the latter mechanism by reducing the concentration of the antibiotic in the target site, thus generating less susceptibility of the bacteria to the compound [11]. The presence of efflux pumps contribute to the resistance towards different antibiotics class, particularly imipenem and tigecycline [12]. Given the importance of efflux pumps in the development of resistance mechanisms by *A*. *baumannii*, efflux pump inhibitors have been widely tested against this pathogen. One of these compounds is carbonyl cyanide 3-chlorophenylhydrazone (CCCP) an uncoupler of oxidative phosphorylation which disrupts the ionic gradient of bacterial membranes [13]. This inhibitor compound has been effectively used in addition to tigecycline to improve susceptibility to this antibiotic [14]. Due to the increasing rates of resistance of *A*. *baumannii* against cefepime and imipenem in the last years [15], the aim of this study was to evaluate the effect of the inhibitor carbonyl cyanide 3-chlorophenylhydrazone (CCCP) on the antimicrobial action of imipenem and cefepime on clinical strains of *A*. *baumannii*.

## Materials and methods

### Clinical samples and bacteria isolates

A total of 49 non-duplicate clinical samples were collected during January through December of 2018 from patients hospitalized in the *Hospital Regional Docente de Cajamarca*. The identification of *A*.*baumannii* was carried out by standard biochemical methods proposed by Bouvet and Grimont [16]. The bacteria isolated were later cultivated in 2mL of trypticase soy agar (TSA) and incubated at 37°C for 18–24 hours. The samples were transported to the molecular biology laboratory of the Universidad Peruana de Ciencias Aplicadas (UPC), where bacterial isolates were reactivated. Of the 49 samples obtained, the confirmatory identification of *A*. *baumannii* was performed on 47 samples by molecular methods previously described [17].

### Amplification of the bla*OXA-51-like gene*

After molecular identification, the amplification of the bla*OXA-51-like gene* was carried out by polymerase chain reaction (PCR). Firstly, DNA extraction was performed using an in-house assay previously reported by Oh et al [18]. Primers and probes used for the molecular identification of the bla*OXA-51-like* gene were previously described by Hu et al. [19]. A commercial strain of *A*.*baumannii* (ATCC 19606) was used as a positive control. Samples were sent for sequencing in Macrogen (Seoul, Korea).

For the detection of genetic material we performed a real-time PCR assay using the *LightCycler 2*.*0 (Roche Diagnostic*, Basel, Switzerland). Conditions used were previously described by Yang et al. [20]: initial 10 minutes at 95 ° C, followed by 55 cycles consisting of: denaturation at 95 ° C for 5 seconds, hybridization at 60 ° C for 5 seconds and elongation at 72 ° C for 15 seconds. Subsequently, we proceeded with the melting curve protocol, which was applied under the conditions of 95 ° C for 20 seconds and then increase of 0.2 ° C / second were executed between 40 ° C to 85 ° C. Data acquisition was obtained during the hybridization stage and in each temperature increase of the melting curve.

### Antibiotic susceptibility profile

The determination of the minimum inhibitory concentration (MIC) was calculated using the microdilution method in culture broth according to the guidelines established in the guide M07-A10 of the Clinical and Laboratory Standard Institute (CLSI) [21], using the following antibiotics: imipenem and cefepime. For the susceptibility assay two groups were formed, to which 240 μL of the bacterial inoculum was added in sterile 1.5 ml tubes. The inoculum was incubated in a shaker at 37 ° C for 18 hours. Posteriorly, the turbidity of the inoculum was adjusted to a 0.5 McFarland standard. One group received 48 μL of free water and the other group received 48 μL of inhibitor.

The antibiotics were serially diluted in Mueller-Hinton (MH) broth in 10 Falcon tubes of 15 mL, obtaining the following concentrations: 256 μg / ml, 128 μg / ml, 64 μg / ml, 32 μg / ml, 16 μg / ml, 8 μg / ml, 4 μg / ml, 2 μg / ml, 1 μg / ml, 0.5 μg / ml, and 0.25 μg / ml. For the experiment, 96-well microplates were used, 90 μl were of antibiotic dilution and 10 μl of bacterial inoculum were added to each well, with a final volume of 100μl. The plates were incubated at 37 ° C for 18 to 24 hours and, after that, the reading was carried out in a spectrophotometer with a 630mm filter.

According to the M100 guide of the CLSI 2020 [22], the cut-off values considered in this study for cefepime were: ≤ 8 (Sensitive), 16 (Intermediate), ≥ 32 (Resistant) and for imipenem: ≤ 2 (S), 4 (I), ≥ 8 (R). For the quality control of microdilution in broth for both antibiotics, Escherichia coli (ATCC^®^ b 25922) and *Pseudomona aeruginosa* (ATCC^®^ b 25922) were used.

Finally, the minimum inhibitory concentration was compared with the reference tables provided by the CLSI instructions M100 [22].

### Addition of the efflux pump inhibitor: Carbonyl cyanide 3 chlorophenylhydrazone (CCCP)

The susceptibility to both antibiotics (cefepime and imipenem) was evaluated in the presence and absence of the inhibitor carbonyl cyanide 3-chlorophenylhydrazone (CCCP) (Sigma–Aldrich, St Louis, MO, USA). Firstly, antibiotics with a concentration ranging from 0.25 a 256 μg/ml was added to each plate containing Muller Hinton broth. After that, CCCP was added to the corresponding plate to a final volume of 100 μl. MIC for each antibiotics was calculated in the presence and absence of the inhibitor CCCP. A 4-fold or greater reduction in the MIC values after the addition of CCCP was considered as a criterion of significance, as proposed by previous authors [23–25]

### Ethics statement

This study was approved by the Research Ethics Board of the *Universidad Peruana de Ciencias Aplicadas*, *Lima*, *Peru* (Document N° CIE/257-10-19). All methods were performed in accordance with the relevant guidelines and regulation. This study was performed on clinical laboratory isolates. The authors had no contact or interaction with the patients. Personal information of the patients was not collected, to guarantee anonymity and confidentiality.

## Results

A total of 49 clinical strains of *A*. *baumannii* were isolated from different hospitalized patients in the Hospital Regional de Cajamarca, of which 47 strains were identified by molecular methods. Table 1 shows the MIC for both antibiotics before and after the addition of the CCCP inhibitor. Based on the MICs obtained, the *A*. *baumannii* strains were classified as susceptible, intermediate, or resistant, according to the cut-off point established by the CLSI for both antibiotics [22]. It can be observed in Fig 1 the susceptibility and resistance patterns according to each antibiotic with and without addition of CCCP. Most of the isolates of *A*. *baumannii* were resistant to both antibiotics tested. Specifically, 97.87% (46/47) of strains were resistant to imipenem, 2.13% (1/47) of them were classified as intermediate and none of these strains were susceptible. On the other hand, 51.06% (24/47) of isolates were resistant to cefepime; 19.15% (9/47) intermediate and 29.79% (14/47) susceptible. With the addition of CCCP it can be observed that resistance patterns changed. In the case of imipenem + CCCP (43/47) were resistant, (2/47) intermediate and (2/47) susceptible. In the case of cefepime + CCCP, (16/47) were resistant, (11/47) intermediate and (20/47) susceptible.

**Fig 1:** Antibiotic susceptibility pattern for each antibiotic before and after addition of CCCP.

**Table 1:** MIC values of cefepime and imipenem against isolated strains of *A*. *baumannii* with and without CCCP addition.

Strain	MIC (μg/ml) for each antibiotic			
	IMIPENEM		CEFEPIME	
	ABX	ABX+ CCCP	ABX	ABX + CCCP
Acc1	32 (R)	64 (R)	16 (I)	8 (S)
Acc2	64 (R)	128 (R)	128 (R)	≥256 (R)
Acc3	128 (R)	64 (R)	32 (R)	≥256 (R)
Acc4	64 (R)	32 (R)	8 (S)	16 (I)
Acc5	64 (R)	8 (R)	64 (R)	8 (S)
Acc6	128 (R)	128 (R)	64 (R)	128 (R)
Acc7	64 (R)	128 (R)	2 (S)	8 (S)
Acc8	64 (R)	64 (R)	16 (I)	4 (S)
Acc9	64 (R)	32 (R)	64 (R)	16 (I)
Acc10	64 (R)	32 (R)	128 (R)	≥256 (R)
Acc11	64 (R)	128 (R)	64 (R)	16 (I)
Acc12	32 (R)	8 (R)	128 (R)	16 (I)
Acc13	32 (R)	8 (R)	32 (R)	8 (S)
Acc14	64 (R)	32 (R)	64 (R)	16 (I)
Acc15	128 (R)	32 (R)	64 (R)	16 (I)
Acc16	16 (R)	32 (R)	64 (R)	4 (S)
Acc17	16 (R)	32 (R)	8 (S)	16 (I)
Acc18	64 (R)	16 (R)	16 (R)	4 (S)
Acc19	128 (R)	64 (R)	≥256 (R)	128 (R)
Acc20	16 (R)	64 (R)	64 (R)	64 (R)
Acc21	8 (R)	4 (I)	64 (R)	64 (R)
Acc22	32 (R)	8 (R)	16 (I)	64 (R)
Acc23	64 (R)	32 (R)	32 (R)	8 (S)
Acc24	4 (I)	0.25(S)	64 (S)	0.25 (S)
Acc25	64 (R)	16 (R)	8 (S)	2 (S)
Acc26	128 (R)	128 (R)	4 (S)	2 (S)
Acc27	64 (R)	16 (R)	2 (S)	0.5 (S)
Acc28	64 (R)	32 (R)	64 (R)	64 (R)
Acc29	64 (R)	128 (R)	8(S)	64 (R)
Acc30	32 (R)	64 (R)	128 (R)	64 (R)
Acc32	64 (R)	64 (R)	8 (S)	1 (S)
Acc33	64 (R)	64 (R)	16 (I)	8 (S)
Acc34	64 (R)	32 (R)	64 (R)	2 (S)
Acc35	64 (R)	32 (R)	2 (S)	4 (S)
Acc36	64 (R)	16 (R)	8 (S)	2 (S)
Acc37	16 (R)	16 (R)	4 (S)	64 (R)
Acc38	16 (R)	2 (S)	64 (R)	128 (R)
Acc39	16 (R)	32 (R)	16 (I)	16 (I)
Acc41	128 (R)	32 (R)	128 (R)	16 (I)
Acc42	64 (R)	32 (R)	32 (R)	32 (R)
Acc43	64 (R)	32 (R)	8 (S)	0.25 (S)
Acc44	64 (R)	64 (R)	16 (I)	4 (S)
Acc45	64 (R)	8 (R)	64 (R)	16 (I)
Acc46	64 (R)	16 (R)	16 (I)	16 (I)
Acc47	64 (R)	32 (R)	16 (I)	64 (R)
Acc48	32 (R)	4 (I)	16 (I)	8 (S)
Acc49	32 (R)	32 (R)	8 (S)	2 (S)

MIC: Minimum inhibitory concentration.

Acc1-49: *A*.*Baumannii* clinical strains, Acc31 and Acc40 were excluded.

(R):Resistant; (I):Intermediate; (S):Susceptible; N/C: no changes.

ABX: Antibiotic.

CCCP: Inhibidor Carbonyl Cyanide m-Chlorophenylhydrazone.

Our comparative analysis shows that the addition of the inhibitor decreased the MIC of imipenem and cefepime as shown in Fig 2. A fourfold or greater reduction in the MIC was used as the criterion for significance. In the case of CCCP in addition to imipenem, 2.1% (1/47) had a significant change of 4 or more reductions in MIC, 59.6% (28/47) achieved a change equal or less than 3 dilutions and 17.0% (8/47) did not have any change. In the case of CCCP with cefepime the percentage of strains with the significant change of MIC was 8.5% (4/47). On the other hand, 53.2% (24/47) presented a reduction equal or less than 3 dilutions and 12.8% (6/47) did not show changes.

**Fig 2:** Reductions in MIC concentration for each antibiotic in combination with the CCCP inhibitor.

## Discussion

In early 2019, the World Health Organization (WHO) published a list of the ten most serious threats to public health, including antibiotic resistance as one of the most important among them [6]. *Acinetobacter baumannii* is a gram-negative coccobacillus implicated in a variety nosocomial infections, with increasing rates of antibiotic resistance. Its ability to survive during long periods of time in hospital settings and its resistance to different antibiotic classes are the main factors implicated in outbreaks caused by this pathogen. This can be observed in our study, in which we found high rates of antibiotic resistance among the 47 samples isolated from the Hospital Regional Docente de Cajamarca, with 46 strains resistant to imipenem and 24 to cefepime.

Efflux pumps are one of the most important mechanisms of antibiotic resistance displayed by *Acinetobacter baumannii*. The overexpression of efflux pumps are associated with a decreased concentration of antibiotics at their target site and an increase in the minimum inhibitory concentration (MIC) [26]. The inadequate use of antibiotics may contribute to the development of efflux pumps and reduce available treatment options [27]. Moreover, antibiotics abuse may be considered one of the most important factors inducing mulidrug-resistance in *A*. *baumannii*. In the current study 97.87% of the strains were resistant to imipenem and 51.06% to cefepime. Gholami et al [23] established that resistance rates of *A*. *baumannii* strains of hospitalized patients in Iran were between 76% to 100% according to the antibiotic tested, nonetheless, all strains were susceptible to colistin. In this study rates of resistance to cefepime and imipenem were 100% and 97%, respectively. There are previous studies in Peru reporting resistance rates of *A*. *baumannii* to different antibiotics. Similar to our study, Levy-Blitchtein et al. [28] demonstrated that 97.5% of *A*. *baumannii* strains isolated in a hospital in Lima, Peru were resistant to carbapenems. In the year 2002, the National Institute of Health of Peru found that resistance rates for *A*. *baumannii* were the highest for amikacin and ceftazidime, and the lowest for carbapenems [29]. Another study performed in Peru by García Rivera et al. [30] evidenced that 93% of strains were resistant to cefepime and 95% to trimethoprim-sulfamethoxazole.

The role of efflux pumps in biofilm formation and antibiotic resistance has been greatly studied in gram negative pathogens. These pathogens are the most common causes of nosocomial infections, resulting from their inherent ability to develop resistance, and are rapidly becoming one of the greatest challenges in modern medicine. The presence of efflux pumps has rendered a variety of bactericides ineffective against *A*. *baumannii* [31]. For example, it has been reported that the presence of efflux pumps corresponding to the resistance-nodulation-cell division (RND) family are an important in resistance to several antibiotic families, including beta-lactams, chloramphenicol, carbapenems, macrolides, tetracyclines, and aminoglycosides [32].

The development of efflux pumps inhibitors constitutes an important advance in the fight against antibiotic resistance. In the current study we could observe the effect of CCCP on susceptibility to imipenem and cefepime. In the case of imipenem, 46 and 43 strains were resistant before and after CCCP addition. In the case of cefepime, 24 and 16 were resistant before and after CCCP addition. It has been previously demonstrated that efflux pumps inhibitors decrease rates of multi-drug resistance in *A*. *baumannii* and other gram-negative bacteria [33, 34]. Particularly, the use of CCCP has been studied previously with optimal results, for example Rjamohan et al [35] reported that adding CCCP reduced the MIC of various biocides by 2 to 12 fold compared to their initial MIC. Likewise, another study performed by Lin et al [36] reported similar effects with the addition of CCCP to ciprofloxacin. In our study, the addition of the CCCP inhibitor decreased resistance in 11 clinical strains. We could observe that initially 0 and 14 strains were susceptible to imipenem and cefepime, respectively. After the use of CCCP in combination with the antibiotics, 2 and 20 strains were susceptible to imipenem and cefepime, respectively.

We observed that only 1 (2.1%) strain achieved the fourfold or greater reduction in MIC for imipenem and 4 (8.5%) strains for cefepime. More than 50% of the strains reduced their MIC by 2–3 dilutions for both drugs. Interestingly, approximately 20% of the strains increased their MIC for both antibiotics by 2–3 dilutions. Other studies report greater reductions in MIC with the use of efflux pumps inhibitors. For example, Gholami et al [23] report that the use of Phenylalanine-Arginine β-Naphthylamide (PAβN) resulted in a 4–64 fold reduction in the MIC for 58 of 60 (96.6%) isolates of *A*. *baumannii*. Similarly, Ardebili and colleagues [13] found that susceptibility of *A*. *baumannii* to ciprofloxacin was highly increased in the presence of CCCP, with 86.1% of their isolates showing MIC reductions by 2 to 64 dilutions. Our findings could be explained by the overall greater resistance at baseline found in our study, nearly all our isolates were resistant to imipenem and more than the half to cefepime. Also, efflux pumps are one of the mechanisms but not always the only mechanism of antibiotic resistance. Several mechanisms are involved in antibiotic resistance in *A*. *baumannii*, such as β-lactamases production, decreased membrane permeability and altered target site of the antibiotic [37–39]. In the present study, the susceptibility to imipenem and cefepime could be greatly affected by the presence of beta lactamases and imipenemases, which are not targeted by efflux pump inhibitors [38]. Finally, we observed a paradoxical effect in some isolates, with an increase in the MIC when CCCP was added. Similarly, Ferrer-Espada et al [40] found that the inhibitor PAβN resulted in a paradoxical effect on bacterial inhibition. This phenomenom has been described as the “Eagle effect”, which results in a paradoxical reduced killing of microorganisms by antibiotics at concentrations higher than their optimum bactericidal concentration [41].

The most important limitation of this study is the lack of information regarding medical records. It would be interesting to analyze the clinical information of the patients, including clinical status, co-morbidities and previous antibiotic use. Also, information of the origin of the samples (biopsies, tissues or secretions) would be essential.

In conclusion our results demonstrate that the use of CCCP may improve *in vitro* susceptibility of *A*. *baumannii* to imipenem and cefepime. The relevance of this study is that it provides evidence that this efflux pump inhibitor may be used in combination with antibiotic therapy, given that pathogens such as *A*. *baumannii* develop intrinsic resistance mechanisms that have rendered most antimicrobial treatments useless. Further studies are required to evaluate the effect of this inhibitor in combination with other antimicrobials, as well as, its effect against other microorganisms. Moreover, CCCP should be studied in the next years to evaluate its *in vivo* activity, as well as, possible adverse effects.
